The article "Protective Effect of Targeted Fluid Therapy on Patients with One-Lung Ventilation" was retracted in 2023. Reasons: signs of a paper mill; compromised peer review; unreliable results or conclusions.

# Protective Effect of Targeted Fluid Therapy on Patients with One-Lung Ventilation

**DOI:** 10.1155/2022/7850031

**Published:** 2022-05-06

**Authors:** Ji-bo Zhao, Yuan-li Li, Deng-Yun Xia, Xiao-Jia Sun, Fu-Long Li, Zhen Xing

**Affiliations:** ^1^Department of Anesthesia, The First Affiliated Hospital of Hebei North University, Zhangjiakou 075000, Hebei, China; ^2^Department of Critical Medicine, The First Affiliated Hospital of Hebei North University, Zhangjiakou 075000, Hebei, China

## Abstract

**Objective:**

To evaluate the protective effect of target-directed fluid therapy on the lungs and postoperative rehabilitation in elderly patients with single-lung ventilation undergoing total endoscopic radical resection of esophageal cancer.

**Methods:**

Seventy elderly patients who underwent total endoscopic radical resection of esophageal cancer from January 2017 to December 2019 in our hospital were selected and divided into two groups by the random number table method: the goal-directed fluid treatment group (group *G*, *n* = 35) and the control group (group *C*, *n* = 35). Venous blood was extracted before surgery (*T*1), at the end of free esophagus (*T*2) by thoracoscopy, at the end of abdominal surgery (*T*3), and at the end of surgery (*T*4). IL-6 and IL-10 levels were detected by ELISA. The clinical pulmonary infection score (CIPS) was used to evaluate the pulmonary inflammation on the second day after surgery and the occurrence of complications. Duration of antibiotic use and length of hospital stay were recorded.

**Results:**

At *T*1, there were no significant differences in IL-6 and IL-10 levels between the two groups (*P* > 0.05). At *T*2, the IL-6 level in group *G* increased to 26.65 ± 1.80 pg/ml but was significantly lower than that in group *C* (32.28 ± 3.22 pg/ml) (*P* < 0.01). At *T*3 and *T*4, IL-6 and IL-10 levels in group *G* were significantly lower than those in group *C* (*P* < 0.01). The CIPS score of group *G* was lower than that of group *C* (1.5 ± 1.0 vs 2.7 ± 1.4), and the duration of antibiotic use in group *G* was shorter than that in group *C* (211.2 ± 15.4 vs 232.6 ± 18.7 h), with statistical significance (*P* < 0.01). The incidence of complications in group *G* was lower than that in group C (28.6% vs 40.0%), and the length of hospital stay in group *G* was shorter than that in group C (10.5 ± 1.7 vs 11.2 ± 1.9 days), but there was no significant difference between the two groups (*P* > 0.05).

**Conclusion:**

Target-directed fluid therapy inhibited inflammatory cytokine levels and had better lung protection, but no significant benefit in the complications or the length of hospital stay was observed.

## 1. Introduction

With the rapid development of minimally invasive technology in recent years, total endoscopic resection of esophageal cancer has become an important minimally invasive surgical method for elderly patients with esophageal cancer [1]. It is worth noting that intraoperative stress and postoperative pulmonary complications caused by single-lung ventilation in such patients are important factors affecting the rapid postoperative recovery of patients [2]. Target-directed fluid therapy is a new concept of perioperative fluid management based on the fluctuation of intraoperative hemodynamic indexes. Compared with the traditional liquid therapy, this method can carry out individualized fluid replenishment according to the circulation status, avoiding not only the fluid overload caused by a large amount of infusion but also the insufficient volume caused by limited infusion [3]. Previous studies have shown that target-directed fluid therapy can improve the patient's microcirculation perfusion, arterial oxygenation, and tissue oxygen supply [4]. This study aims to evaluate the protective effect of goal-directed fluid therapy on the lungs and its influence on postoperative rehabilitation in elderly patients undergoing single-lung ventilation during total endoscopy radical resection of esophageal cancer, so as to provide some theoretical reference for clinical treatment.

The article "Protective Effect of Targeted Fluid Therapy on Patients with One-Lung Ventilation" was retracted in 2023. Reasons: signs of a paper mill; compromised peer review; unreliable results or conclusions.

## 2. Materials and Methods

Seventy elderly patients with ASA I-II grade were selected for total endoscopic radical resection of esophageal cancer from January 2017 to December 2019 in our hospital. The inclusion criteria were patients over 65 years of age with basal heart rate >60 beats/min and forced expiratory volume in the first second (FEV1) ≥70% of the estimated value. The exclusion criteria were long-term use of sedative-hypnotic or antipsychotic drugs before surgery; complications with serious heart, liver, lung, and kidney diseases; and patients with severe postoperative complications such as esophagotracheal fistula, thoracic duct injury, and chylothorax. All patients strictly quit smoking and underwent respiratory exercise before surgery. Seventy patients were divided into two groups using the random number table method: the target-directed fluid treatment group (*G* group, *n* = 35) and the control group (*C* group, *n* = 35). All patients or their authorized family members signed informed consent, and the protocol of this study was approved by the Ethics Review Committee of The First Affiliated Hospital of Hebei North University.

### 2.1. Intraoperative Management and Data Collection

Target-directed fluid treatment group *G* [5] used a MostCare monitor to monitor the stroke volume variation (SVV) and cardiac index (CI) for fluid replenishing. Before induction of anesthesia, 5–7 mL/kg of 6% hydroxyethyl starch was infused intravenously, followed by a continuous infusion of compound sodium lactate Ringer's solution at 8 mL/(KGXH). If SVV ≤11% and CI >2.5 L/(Minxm2), the original solution was continued for infusion. If SVV >11%, an intravenous infusion of 50 mL/min of 6% hydroxyethyl starch solution was administered until SVV ≤11% for more than 2 minutes. Control group *C* received classical fluid therapy. The patient's demographic data, physical examination, and lung function data were collected, and the operation time, single-lung ventilation time, and anesthesia time were recorded. Venous blood was extracted before surgery (*T*1), at the end of free esophagus (*T*2), at the end of abdominal surgery (*T*3), and at the end of global surgery (*T*4), and IL-6 and IL-10 concentrations were detected by ELISA. The pulmonary infection score was used to evaluate the pulmonary inflammation on the second day after surgery, and the occurrence of complications was recorded according to the POMS scale [6], and the duration of antibiotic use and hospital stay were recorded.

The article "Protective Effect of Targeted Fluid Therapy on Patients with One-Lung Ventilation" was retracted in 2023. Reasons: signs of a paper mill; compromised peer review; unreliable results or conclusions.

### 2.2. Statistical Analysis

All statistical analysis was performed by the SPSS 21.0 statistical software. Continuous variables were expressed by (x ± s) and compared by the *t*-test. Categorical variables were expressed as a percentage (n (%)) and compared by the Chi-square test. *P* < 0.05 was used to assess statistical significance.

## 3. Results

### 3.1. Comparison of General Data and Intraoperative Indicators

As shown in Table 1, the age of patients in group *G* was 74.0 ± 5.5 years old, the male proportion was 62.9%, the average BMI was 24.3 ± 2.5, and FEV1/FVC was 80.4 ± 7.2%. The operation time, single lung ventilation time, and anesthesia time of group *G* were 235 ± 40, 182 ± 40, and 268 ± 41 min, respectively. There were no statistically significant differences between group *G* and group *C* in age, sex ratio, ASA grading ratio, BMI, FEV1/FVC, operation time, single lung ventilation time, and anesthesia time (*P* > 0.05).

### 3.2. Comparison of IL-6 and IL-10 Levels at Different Time Points

As shown in Table 2, there was no significant difference in the IL-6 level between group *G* and group *C* at *T*1 (*P* > 0.05). At *T*2, the IL-6 level in group *G* increased to 26.65 ± 1.80 pg/ml but was significantly lower than that in group *C* (32.28 ± 3.22 pg/ml) (*P* < 0.01). At *T*3 and *T*4 time points, the IL-6 level in group *G* was still significantly lower than that in group *C* (*P* < 0.01). There was no significant difference in the IL-10 level between the two groups at *T*1 (*P* > 0.05). At *T*2, the level of IL-10 in group *G* increased to 30.75 ± 4.59 pg/ml but was significantly lower than the level of IL-6 in group *C* (35.36 ± 2.89 pg/ml) (*P* < 0.01). At *T*3 and *T*4 time points, the IL-10 level in group *G* was still significantly lower than that in group *C* (*P* < 0.01).

The article "Protective Effect of Targeted Fluid Therapy on Patients with One-Lung Ventilation" was retracted in 2023. Reasons: signs of a paper mill; compromised peer review; unreliable results or conclusions.

### 3.3. Comparison of CIPS Score, Duration of Antibiotic Use, Incidence of Complications, and Length of Hospital Stay

The CIPS score of group *G* was lower than that of group *C* (1.5 ± 1.0 vs 2.7 ± 1.4), and the duration of antibiotic use in group *G* was shorter than that in group *C* (211.2 ± 15.4 vs 232.6 ± 18.7 h), the differences were statistically significant (*P* < 0.01). The complication rate in group *G* was lower than that in group *C* (28.6% vs 40.0%), and the length of hospital stay in group *G* was shorter than that in group *C* (10.5 ± 1.7 vs 11.2 ± 1.9 days), but there was no significant difference between the two groups (*P* > 0.05) (Table 3).

## 4. Discussion

We found that patients in the goal-directed fluid treatment group *G* had lower IL-6 and IL-10 levels, lower lung infection scores (CIPS), and shorter duration of antibiotic use in elderly patients undergoing single-lung ventilation after total endoscopy for esophageal cancer compared with those of control group *C*. There also seemed to be a tendency for fewer complications and shorter hospital stays in group *G*.

Total endoscopic esophageal cancer surgery is becoming advanced and is being gradually promoted due to its advantages of minimally invasive surgery and thorough lymph node dissection [7]. However, intraoperative lung injury and postoperative lung infection are common complications in elderly patients with esophageal cancer and are the leading cause of perioperative death [8]. Factors affecting lung injury and lung infection mainly include hyperactivity of oxygen free radicals and inflammatory response, and the single-lung ventilation process during surgery can lead to the release of various cytokines, thus triggering systemic inflammatory response [9]. IL-6 and IL-10, as markers of tissue damage, are significantly correlated with the degree of surgical trauma and inflammatory response, as well as postoperative recovery of patients [10]. In this study, target-directed fluid therapy was found to be associated with a decrease in IL-6 and IL-10 levels, suggesting that target-directed fluid therapy may help suppress excessive inflammatory responses. As a relatively new concept, target-directed fluid therapy aims to optimize the cardiac preload through individualized fluid replenishing strategies, maintain effective circulating blood volume and oxygen supply, avoid tissue edema and tissue hypoxia, and thus improve postoperative recovery [11]. It is very important to select appropriate hemodynamic parameters in target-directed fluid therapy. SVV is the main dynamic parameter guiding the target-directed fluid therapy. SVV has high sensitivity and specificity in the fluid therapy of patients with single-lung ventilation and can accurately evaluate the patient volume status [12]. This study found that patients in the target-directed fluid treatment group had lower pulmonary infection scores and shorter duration of antibiotic use. This may be attributed to the following factors: (1) target-directed fluid therapy reduces the possibility of ischemic lung injury by maintaining an effective circulating blood volume and oxygen supply [13]; (2) target-directed fluid therapy, by inhibiting inflammatory overreaction, promotes the recovery of the patient's systemic state and reduces the possibility of lung infection, thus shortening the time of antibiotic use [14]; (3) in the process of target-directed fluid therapy, medical staff are more careful in the treatment monitoring and nursing process of patients and timely detect the changes in their condition, which may also bring therapeutic benefits [15]. However, it is worth noting that this study also found that the patients in the target-directed fluid treatment group also seemed to have a tendency to reduce complications and shorten the length of hospital stay, partly due to the limited sample size of our study. In addition, the reasons to be analysed may be that the return of patients to the ward after surgery, the occurrence of complications, and the length of hospital stay are affected by a variety of factors, such as the factors of nursing staff and the factors of patient's families. In the future, we will need larger sample sizes to better control for possible confounders between the two groups to further clarify the benefits of target-directed fluid therapy. In conclusion, patients in the target-directed fluid treatment group had lower IL-6 and IL-10 levels, lower lung infection scores (CIPS), and shorter duration of antibiotic use when undergoing single-lung ventilation after total endoscopic radical resection of esophageal cancer, but no significant benefit was found in reducing complications and shortening the length of hospital stay.

The article "Protective Effect of Targeted Fluid Therapy on Patients with One-Lung Ventilation" was retracted in 2023. Reasons: signs of a paper mill; compromised peer review; unreliable results or conclusions.

## Figures and Tables

**Table 1:** Comparison of general data and intraoperative indicators (*n* = 70).

Group	Age	Male, *n* (%)	ASA grade ratio (I/II)	BMI, kg/m^2^	FEV1/FVC, %	Operationtime, min	One-lung ventilation time, min	Anesthesiatime, min
Group *G* (*n* = 35)	74.0 ± 5.5	22 (62.9)	16/19	24.3 ± 2.5	80.4 ± 7.2	235 ± 40	182 ± 40	268 ± 41
Group C (*n* = 35)	72.6 ± 5.9	21 (60.0)	15/20	24.7 ± 4.1	79.9 ± 7.1	221 ± 39	169 ± 40	257 ± 41

**Table 2:** Comparison of IL-6 and IL-10 levels at different time points.

Group	*T*1	*T*2	*T*3	*T*4
*IL-6 (pg/ml)*				
Group *G* (*n* = 35)	4.99 ± 0.92	26.65 ± 1.80^*∗*^	28.39 ± 2.92^*∗*^	29.67 ± 3.12^*∗*^
Group *C* (*n* = 35)	5.16 ± 1.26	32.28 ± 3.22	33.56 ± 3.73	34.20 ± 3.76

*IL-10 (pg/ml)*				
Group *G* (*n* = 35)	9.95 ± 1.37	30.75 ± 4.59^*∗*^	33.21 ± 4.67^*∗*^	34.70 ± 4.62^*∗*^
Group *C* (*n* = 35)	10.29 ± 1.48	35.36 ± 2.89	37.50 ± 3.21	38.55 ± 3.36

^*∗*^Compared with group *C*, *P* < 0.01.

**Table 3:** Comparison of CIPS score, duration of antibiotic use, the incidence of complications, and the length of hospital stay.

Group	CIPS scores	Antibiotic use time, h	Complication rate, *n* (%)	Length of stay, days
Group *G* (*n* = 35)	1.5 ± 1.0^*∗*^	211.2 ± 15.4^*∗*^	10 (28.6)	10.5 ± 1.7
Group *C* (*n* = 35)	2.7 ± 1.4	232.6 ± 18.7	14 (40.0)	11.2 ± 1.9

^*∗*^Compared with group *C*, *P* < 0.01.

## Data Availability

The data used to support the findings of this study are available from the corresponding author upon request.
